The article "Analysis of the Effect of Percutaneous Cone Shaping in Patients with Osteoporotic Vertebral Fractures" was retracted in 2023. Reasons: signs of a paper mill; suspected computer-generated content; unreliable results or conclusions; lack of ethics approval or compliance.

# Analysis of the Effect of Percutaneous Cone Shaping in Patients with Osteoporotic Vertebral Fractures

**DOI:** 10.1155/2022/5188703

**Published:** 2022-08-09

**Authors:** Jiasheng Yu, Daobo Fan, Lei Bao, Dongqian Feng, Bin Zhang

**Affiliations:** Department of Orthopedics, Shuyang Hospital of Traditional Chinese Medicine, Clinical College of Yangzhou University Medical College, Yangzhou, China

## Abstract

**Objective:**

To study and analyze the clinical effect of percutaneous cone shaping in patients with osteoporotic vertebral fractures.

**Methods:**

A total of 100 patients with vertebral osteoporotic fracture treated in our hospital from June 2019 to September 2020 were selected, and there were 50 patients with vertebral osteoporotic fracture in each group. Patients could be divided into two groups according to different treatment plans: one group was vertebroplasty patients for group A, and the other group was nonsurgical treatment patients for group B. The incidence of complications during treatment and follow-up was recorded in both groups.

**Results:**

According to a study, both groups of patients completed the treatment and follow-up, no patients lost to follow-up or death, the VAS scores and ADL scores of patients before treatment were higher, and there was no significant difference at baseline (*P* > 0.05). After different treatment methods, the VAS score and ADL score of group A showed good improvement after treatment compared with that before treatment, and there were certain differences within the group, with statistical significance (*P* < 0.05). Intragroup comparison. The VAS scores of group B at 1 week, 1 month, 3 months, and 12 months after treatment were all superior to those before treatment, and the ADL scores at 1 month, 3 months, and 12 months after treatment were all superior to those before treatment, with statistically significant differences (*P* < 0.05). VAS scores and ADL scores showed good improvement 1 day, 1 week, and 1 month after treatment compared with those before treatment. However, there were no significant differences in the VAS score and ADL score between the two groups at 3 and 12 months after treatment. The incidence of complications in group A is lower than that in group B. The incidence of complications in group A is as follows: there was 1 case of recurrent vertebral fracture and 1 case of urinary tract infection, and the overall incidence of complications was 4.00%. In group B, there were 1 case of recurrent fracture, 3 cases of bedsore, 2 cases of urinary tract infection, and 2 cases of pulmonary infection, and the incidence of total complications was 16.00%. After comparison between groups, there was a significant difference in the incidence of complications between the two groups, and the difference was statistically significant (*P* < 0.05).

**Conclusions:**

Percutaneous cone plasty can provide rapid relief of pain symptoms in patients with osteoporotic vertebral fractures and significantly improve their daily activities. However, there was no significant difference in long-term recovery from group B. In terms of the incidence of complications, the incidence of complications in group A was lower than that in group B after certain treatment.

## 1. Introduction

Osteoporosis is a kind of bone disease syndrome caused by many causes [1]. In the normal state of the human body, there will be normal calcification of bone tissue, and the bone matrix and calcium salt will reach a balance state in a certain range. However, with the gradual increase in the human age, bone absorption will gradually increase, resulting in a sharp decline in the amount of bone tissue in the same unit volume, resulting in a series of metabolic bone diseases; the main feature is the occurrence of osteoporosis, which is a common disease in the elderly [1]. After the occurrence of osteoporosis to a certain extent, elderly patients will be affected due to less calcium salt deposition in bone and bone strength and toughness will be significantly decreased [2]. In the elderly patients, especially the lumbar vertebral compression fracture is more common, and the main reason for most patients to seek medical treatment is because of pain [3]. In general, patients with bone loss of more than 12% can develop systemic bone pain, and thoracolumbar compression fractures can be accompanied by acute or severe back pain. Due to the severity of fracture, some patients have been compressed to the spinal nerves, which can also cause sensory motor disorders of lower limbs, radioactive pain in limbs, and pain behind the sternum. Once the patient's spinal cord or cauda equina nerve is compressed, it can also affect the function of the rectum or bladder to a certain extent. Therefore, the occurrence of osteoporosis will seriously affect the quality of life of elderly patients [4]. With the acceleration of the aging of the population, the proportion of osteoporosis is increasing year by year, which indirectly leads to the increase of the incidence of osteoporotic spinal compression fracture, and the thoracolumbar vertebral body is the most common spine fracture due to the large load bearing. Osteoporotic vertebral compression fracture refers to the gradual loss of vertebral bone tissue due to osteoporosis, resulting in the reduction in the bone density and bone strength, which results in single or multiple vertebral compression fractures. Osteoporotic vertebral compression fractures can be diagnosed according to clinical manifestations and auxiliary examination. The main symptoms of patients are low back pain, unable to stand or sit for a long time, and the need to rest in bed. Vertebral compression fractures should be suspected in patients with osteoporosis who present with acute or chronic low back pain, regardless of a history of trauma. X-Ray or CT examination of the corresponding segment can further confirm the diagnosis, MRI examination is necessary, and bone mineral density measurement is feasible for patients with conditions.

The treatment of osteoporotic vertebral compression fracture includes nonoperative treatment and surgical treatment. Nonsurgical treatment includes bed rest, lumbar and back muscle exercises, analgesia, wearing braces, anti-osteoporosis, and other treatments. A specific method includes that when lying on a rigid bed strictly, the spine was repositioned with the aid of analgesic drugs; the patients were instructed to exercise the lumbar and back muscles in bed early after the pain was relieved about 1 week later, the patients were protected to get out of bed 4 weeks later, and the daily activities of the braces were removed 12 weeks later [5]. During the treatment, it can assist to promote blood circulation and fatigue; and promote fracture healing, anti-osteoporosis, and other drug therapies, as well as medium frequency pulse electric therapy, wax therapy, and other physical therapies. Osteoporotic vertebral compression fractures are contraindications for surgical treatment. Surgical treatment should be considered only when the symptoms of spinal cord injury, CT, MRI, and other imaging findings show obvious injury segments, spinal stenosis, and spinal cord compression. Spinal cord compression can be removed by treatment. Internal fixation is generally considered dangerous because it increases fractures of adjacent vertebral bodies and the development of osteoporosis, and in patients with osteoporosis, the lack of vertebral grip on pedicle screws may result in surgical failure. Some surgeons now use modified pedicle internal fixation, that is, the application of internal fixation surgery and pedicle bone cement filling to enhance the pedicle screw control. The clinical manifestations of osteoporosis are not obvious, and the onset is insidious. For most patients, the diagnosis is usually made at the time the fracture occurs [6]. Brittle fractures are nonviolent and occur when there is no obvious force on the bone. Osteoporotic fracture is a local histopathological change based on systemic osteoporosis and is a definite manifestation of reduced bone strength, thus distinguishing it from trauma. Osteoporotic fracture occurs on the basis of osteoporosis, so the incidence of disease is high, the treatment effect is not good, and the rate of death and disability is high. At the same time, because the treatment cycle is relatively long, the effect is poor and the medical cost is significantly higher. Osteoporotic fracture is a bone disease that seriously affects the health of the majority of middle-aged and elderly people. However, the current status of the diagnosis and treatment of osteoporotic fracture in China is really not optimistic, with the phenomenon of delayed diagnosis and systematic treatment. Moreover, different hospitals and doctors have different treatment plans and there is a lack of standardization. Basically, fractures can be divided into two types: compression fracture and burst fracture; compression fracture is more common. Formation of osteoporotic vertebral fracture is the main reason for the patients with osteoporosis; after the body element, progressive loss of bone calcium osteopsathyrosis increases, leading to a great reduction in bone strength and bone mineral density, and thoracic lumbar segment in the thoracic and lumbar spine due to mechanical impact encounters violent shocks, and directly or indirectly, fracture probability is extremely high. However, China's national conditions are that the aging of the population is becoming increasingly serious, resulting in a significant increase in the incidence of osteoporosis, so it has become the focus of our attention. Pain and spine-related dysfunction are typical clinical symptoms of osteoporotic vertebral fractures [7]. When nerves are affected, there is often limited activity, and some are accompanied by other system dysfunction, which has a significant impact on patients' lives. So conservative treatment and surgical treatment are the basic treatment methods. Percutaneous pedicle screw fixation is a common surgical option.

## 2. Data and Methods

### 2.1. General Information

The subjects selected for this study were 100 patients with osteoporotic vertebral fractures treated in our hospital from June 2019 to September 2020, with 50 patients in each group. Patients can be divided into two groups according to different treatment regimens. One group is the patients receiving vertebroplasty, and the other group is the patients receiving nonsurgical treatment. All patients met the criteria for inclusion and exclusion. Of the 100 patients, 49 were women and 51 were men. The average age of the patients in group A was 45.4 ± 4.1 years. The main reasons for the injuries of the patients were as follows: 11 cases of falls, 9 cases of falls, 24 cases of traffic accidents, and 6 cases of patients without significant causes. The disease course of the patients was generally about 0.5 to 3 days. According to the fracture grading, it can be divided into three grades: i degree, 12 cases; ii degree, 23 cases; and iii degree, 15 cases. The average age of the patients in group B was 44.5 ± 4.8 years, and the main reasons for the injuries were as follows: 26 cases of falls, 9 cases of falls, 12 cases of traffic accidents, and 3 cases of patients without significant causes. The disease course of the patients was generally about 0.5 to 3 days. There were 5 cases of grade i, 32 cases of grade ii, and 13 cases of grade iii. There were no significant differences in age, fracture causes, and fracture grades between the two groups (*P* < 0.05).

### 2.2. Inclusion and Exclusion Criteria

#### 2.2.1. Included Criteria

1. Patients with single-stage thoracolumbar compression fractures.
2. X-Ray, CT, or MRI imaging examination showed vertebral compression fracture.
3. Previous spinal activities were basically normal.
4. No lung or urinary tract infection and no obvious low lung function (heart function is better than grade ii patients); ⑥ patients can normally read general words, and the subjective feelings can be described in detail.
5. All patients have been informed of the whole process of the study and can always cooperate with the patients in the study, and all patients have signed informed consent.

#### 2.2.2. Exclusion Criteria

1. Complicated systemic infection has not been effectively controlled.
2. Mental disorders or illiteracy.
3. Severe malnutrition and severe hypoproteinemia, which can seriously affect fracture healing.
4. Pathologic fracture caused by old or bone tumor.
5. Patients with neurological symptoms.
6. Short follow-up time, less than one year.
7. Patients cannot cooperate with the experimenter.
8. Patients with mental diseases who are unable to communicate normally.
9. Patients who cannot recognize and read and write Chinese

### 2.3. Methods

#### 2.3.1. Preparation for Admission

After admission, the patient took absolute bed rest and underwent routine imaging (thoracolumbar X-ray, CT or MRI examination, chest X-ray, electrocardiogram, and related laboratory examination (blood routine, coagulation four items, in-hospital biochemistry, preoperative eight items)) to exclude other benign and malignant spinal lesions. Symptomatic treatment was actively given to the patients with underlying diseases before surgery, among which 5 patients were complicated with diabetes. After consultation with the endocrinology department, “four-needle therapy” of membrane insulin was applied to control blood glucose, and fasting blood glucose was controlled below 9.2 mmol/L. Six patients with hypertension were continued to take usual antihypertensive drugs, and their blood pressure was controlled below 160/100 mmHg. Surgical treatment was performed as soon as the patient's physical condition allowed, and surgery was performed within 2–3 days of admission for patients without other serious complications.

#### 2.3.2. Treatment Methods

Patients in group A were treated in the prone position, with horizontal pads of the anterior superior spine and manubrium sternum to maintain the thoracolumbar overextension position, and the C-arm machine was adjusted to show a first-line shadow of the upper and lower endplates of the vertebral body under orthographic fluoroscopy, which could clearly display the circular projection of the affected vertebrae. The affected vertebrae were accurately located and marked: disinfection towel, 2% lidocaine hydrochloride local infiltration anesthesia, C-arm fluoroscopy guided by the external and upper position of the orthotopic vertebral pedicle (10 : 00 on the left, 2 on the right: 00), and the sagittal plane at an angle of about 15°. When the tip of the needle just entered the posterior, middle, and front of the pedicle, the anteropositive position should show that the needle was located at the lateral wall, midline, and medial edge of the pedicle shadow, respectively, indicating that the direction is correct and the insertion can be continued. When the lateral view shows that the tip reaches the first three quarters of the vertebral body, it is ideal that the tip tilts slightly toward the cephalic side and the inclined plane of the needle head should be toward the midline of the vertebral body. After the completion of the pedicle puncture, the bone cement was prepared, and when the bone cement reached the wire drawing stage, the bone cement was injected into the target vertebra through the established channel under the supervision of the C-arm machine. The injection amount was generally 4–6 ml in the lumbar vertebra and 3-4 ml in the thoracic vertebra. If there was bone cement leakage outside the vertebra, the injection should be stopped immediately. After the cement has hardened completely, remove the puncture needle. Postoperative treatment: adjuvant treatments such as Honghua injection and Lugua Duofu injection were given to promote fracture healing and blood circulation and reduce insanity.

Usually, a single supine position can lead to unbearable patient, prone position can be given discontinuous reduction, the orthopaedic reduction pillow is placed in the chest of the patient, and keep the spine too mid-position. After about 1 week of lumbar back pain relief, patients can be guided to carry out active lumbar back muscle function exercise. In the initial stage, five-point support method can be adopted, that is, flexion of both upper limbs and lower limbs and five-point support of feet, elbows, and head; arch the torso up; and keep the spine overextended. Relax after 3–5 seconds in this position, 50–100 times/day. One week later, imaging examination was performed to observe the vertebral body reduction. After 4 weeks, the patient can move out of bed with the help of a spinal extension brace. After 12 weeks, the brace can be removed for daily life. During the treatment, adjuvant therapies such as Honghua injection and Lugua Duofu injection were given to promote fracture healing and blood circulation and exhaustion.

### 2.4. Observed Indicators

Classification of fracture degree is shown in Table 1.

Before treatment, visual analogue scores of pain and daily living activities were evaluated. VAS score and ADL score were measured again at 1 day, 1 week, 1 month, 3 months, and 12 months after treatment.

VAS score standard is based on the degree of the patient's pain: 0 represents no pain; 10, severe pain; 1–3 points, mild pain— a sustainable state; 4–6, moderate pain—this pain is tolerable, but also affects the patient's normal sleep; and 7 to 10 points, severe pain—intolerable pain and affects the patient's normal sleep and normal diet.

ADL scoring was carried out by the Barthel index after some improvement. Indicators included in the scoring were mainly daily activities, including eating, bathing, rest, dressing, Going to the toilet, transfer, upstairs, and downstairs. As shown in Table 2 that the total score of this score is 100, patients with a score of more than 60 are able to carry out normal activities, indicating that they have the ability to take care of themselves; patients with a score of 40–60 still need help; patients with a score of 20–40 are dependent on others in daily life. In most of life, people are needed to help complete, and patients with less than 20 points indicate that patients have functional defects and are highly dependent on people in life.

### 2.5. Score of Disease

The classification and scoring system of thoracolumbar injury was proposed based on the American spinal trauma study. The scoring system is mainly based on the neurological status of the patient, the structural integrity of the posterior primary band of the affected vertebra, and the mechanism of fracture injury. The specific criteria are as follows: 1. The patient's neurological function status—0 points: no symptoms of neurological damage; 2 points: incomplete spinal cord injury or cauda equina syndrome; and 3 points: complete spinal cord injury. 2. Fracture morphology or fracture mechanism—1 points: compression fracture; 2 points: burst fracture; 3 points: rotary fracture; and 4 points: stretch fracture. 3. The integrity of the composite structure of the posterior primary band of the vertebral body—0 points: the primary band was complete; 2 points: incomplete fracture of primary zone structure; and 3: the primary zone structure is completely fractured; the total TLICS score is calculated by adding the scores.

### 2.6. Statistical Analysis

SPSS 26.0 statistical software was used for the statistical analysis of the data. X2 was used for counting data, and the *T* test was used for the measurement of data. *P* < 0.05 was statistically significant.

## 3. Results

### 3.1. VAS Scores of the Two Groups

Patients in both groups were treated and followed up, and there were no lost patients. There was no significant difference in VAS score and ADL score between the two groups before treatment. As shown in Table 3 that after different treatment methods between the two groups, the VAS score and ADL score of group A showed good improvement after treatment compared with those before treatment, and there were certain differences within the group, with a statistical significance of *P* < 0.05. Within the group, the VAS scores of group B at 1 week, 1 month, 3 months, and 12 months after treatment were better than those before treatment, and the ADL scores at 1 month, 3 months, and 12 months after treatment were better than those before treatment, with statistical significance (*P* < 0.05). Comparison between groups: VAS scores and ADL scores showed good improvement 1 day, 1 week, and 1 month after treatment compared with those before treatment. However, there were no significant differences in VAS scores and ADL scores between the two groups at 3 and 12 months after treatment. A comparison of ADL scores between the two groups is shown in Table 4.

### 3.2. Comparison of the Height of Anterior Vertebral Margin between the Two Groups

As shown in Table 5 that during early treatment and follow-up, the incidence of complications in group A was lower than that in group B, and the incidence of complications in group A was as follows: there were 1 case of recurrent vertebral fracture and 1 case of urinary tract infection, and the overall incidence of complications was 4.00% as shown in Table 6. In group B, there were 1 case of recurrent fracture, 3 cases of bedsore, 2 cases of urinary tract infection, and 2 cases of pulmonary infection, and the incidence of total complications was 16.00%. After comparison between groups, there was a significant difference in the incidence of complications between the two groups, and the difference was statistically significant (*P* < 0.05).

## 4. Discussion

Osteoporosis is a kind of bone disease in which the reduction of bone tissue per unit volume is the main clinical feature caused by various internal or external factors. Normal calcification was observed in bone tissue, and bone matrix was in normal proportion to salt. Reduced bone strength inevitably leads to increased risk of fracture and brittleness [8]. Osteoporosis can be primary or secondary, and about 90% of them are primary. The common primary ones in our life are congenital, senile, and postmenopausal. Because China's national conditions are aging population growth, and now work pressure leads to less exercise, it will inevitably lead to the gradual increase of osteoporosis. Osteoporotic fractures are increasing year by year, bringing serious burden and influence to patients and their families. Compared with normal vertebrae, osteoporotic vertebrae undergo significant changes in bone structure, which is manifested as reduced trabecular bone, thinning of structure, and fracture defect, resulting in enhanced bone fragility [9, 10]. As a result, the osteoporotic vertebral compression fracture is more common in clinical practice than osteoporotic fracture of femoral neck. The clinical symptoms of thoracolumbar compression fractures are more obvious due to pain, and limited movement, severe fracture, and spinal nerve compression can lead to a feeling of lower limb movement disorders, limb pain in radiation, chest pain, and intercostal neuralgia [11]. Compression of the spinal cord and caudal nerves can also affect rectal and bladder function, seriously affecting quality of life. Pain is the most common symptom of primary osteoporosis, and the number one reason patients seek medical attention [12]. It is mainly manifested as systemic bone pain, which is mainly manifested as low back pain. The pain symptoms are aggravated when standing for a long time, bending, coughing, and increasing abdominal pressure. However, in the sitting position and the sitting position, due to the small bone load, the above symptoms can reduce AST. In general, general or local bone pain may occur in the normal population with bone mass loss of more than 12%. For elderly patients, the degree of osteoporosis is generally more serious than that caused by other reasons [13]. The vertebral body strength of patients is significantly reduced, compressive deformation may occur, the spine loses its normal shape, and fatigue and even recovery of the muscles near the spine, such as erector spine, may cause obvious pain symptoms. Vertebroplasty is a new technique that has been applied in clinical practice in recent years. The surgeon injects proper amount of bone cement into the vertebra through percutaneous pedicle or external pedicle in a minimally invasive way to fix the damaged vertebra, which prevents further collapse of the vertebra, so as to increase the stability and strength of the vertebra. The height of the injured vertebral body can be recovered to some extent in some patients. Percutaneous vertebroplasty (PERcutaneous vertebroplasty) is used to treat vertebral compression fractures caused by osteoporosis. After surgery, patients' pain symptoms are effectively relieved; thus, the technique is gradually applied in clinical practice [14].

In the actual treatment, PVP mainly punctures the pedicle and injects filler into the compressed vertebral body to improve the stress intensity of the vertebral fracture, so as to enhance the stability of the spine. Its clinical application effect is good. PVP treatment technology is a microsurgical operation using image guidance to treat vertebral compression fractures. The whole operation process does not need to adopt the way of internal fixation, so it can better retain the motor function of the upper and lower segments, more in line with the characteristics of physiological structure, and achieve the purpose of treatment [15–17]. There are many studies on senile osteoporotic thoracolumbar compression fractures at home and abroad, and all show that the clinical effect of PVP is very significant. In the results of this study, compared with that before treatment, the VAS scores of the two groups decreased significantly after treatment, and the VAS scores of the observation group were significantly lower than those of the control group one week after treatment (*P* < 0.05). After treatment, the height of the anterior edge of the vertebral body, the height of the middle line of the vertebral body, and the Cobb angle of the two groups were significantly improved, and the improvement degree of the observation group was more significant than that of the control group, with statistically significant differences (*P* < 0.05), which further explained the correctness of the above view. Therefore, PVP in the treatment of senile osteoporotic thoracolumbar compression fractures can quickly alleviate the pain of patients and achieve a more ideal treatment effect, which is worthy of clinical application.

The technique, which uses bone cement to fix the injured vertebrae in the early stages of fracture, is effective in relieving pain symptoms, encouraging patients to move out of bed early and improving quality of life.

## 5. Conclusion

In summary, in recent years, domestic and foreign scholars have carried out a large number of clinical and laboratory studies on the treatment of osteoporotic vertebral compression fractures, and relevant research results have been widely applied in clinical practice and achieved some good results. Percutaneous vertebroplasty (PERcutaneous vertebroplasty) is used to treat vertebral fractures caused by osteoporosis. It is effective in relieving pain symptoms after surgical treatment and reducing the incidence of postoperative complications. Percutaneous vertebroplasty (PERcutaneous vertebroplasty) has been shown to improve daily quality of life and long-term outcomes in the treatment of osteoporotic vertebral fractures. It is worth popularizing in clinic.

## Figures and Tables

**Table 1:** Refer to spinal compression fracture scaling.

Dividing	Degree of description
I degrees	The patient had a compression one-third fracture of the cone
II degrees	The patient had a compression half fracture of the cone
III degrees	The patient had a fracture of two-thirds or more of the cone with compression

**Table 2:** ADL scoring criteria.

Project	Score	Situation
Eating	10	Independent eating, the whole process without assistance.
	8	Can eat independently, but special operations such as cutting meat, opening bottle caps, and other actions need assistance
	5	Eat under supervision, but more complex movements require assistance.
	2	Can operate eating tools such as chopsticks, knife, and fork and spoon
	0	Totally dependent on others for food.

Take a shower	10	You can shower independently
	8	Assistance is needed in adjusting the water temperature for timely transfer
	5	Need assistance in cleaning
	2	Every step of the bathing process requires human assistance
	0	Total dependence

The toilet	10	Can independently go to the toilet, and can carry out independent cleaning
	8	It should be carried out under supervision, including the use of urinal at night, with assistance in cleaning
	5	Help with cleaning clothes and washing hands.
	2	Assistance is required at any step of the process.
	0	Total dependence

Up and down the stairs	10	Up and down a flight of stairs.
	8	Up and down a flight of stairs.
	5	Assistance is required when going upstairs and downstairs
	2	Assistance is needed throughout the process.
	0	Don't go upstairs or downstairs.

**Table 3:** VAS scores between the two groups.

Group	Before the treatment	After treatment				
		1 day	1 week	1 months	3 months	12 months
Group A	6.9 ± 3.4	3.2 ± 1.8ab	1.7 ± 2.2ab	1.4 ± l.1ab	l.l ± 0.7a	1.5 ± l.1a
Group B	6.8 ± 3.1	6.7 ± 3.4	5.1 ± 1.6a	2.9 ± 1.6a	1.2 ± 0.6a	1.4 ± 1.2a

*Note.* A refers to the comparison with before treatment, *P* < 0.05. B refers to group B at the same time (*P* < 0.05).

**Table 4:** Comparison of ADL scores between the two groups.

Group	Before the treatment	After treatment				
		1 day	1 week	1 months	3 months	12 months
Group A	67.3 ± 15.4	79.3 ± 1.6^ab^	88.4 ± 2.1^ab^	89.5 ± 0.7^ab^	91.6 ± 1.4^a^	90.5 ± 2.7^a^
Group B	66.7 ± 13	67.3 ± 13.2	73.4 ± 12.7	79.2 ± 1.6^a^	89.4 ± 0.6^a^	89.3 ± 1.7^a^

Note. A refers to the comparison with before treatment, *P* < 0.05. B refers to group B at the same time (*P* < 0.05).

**Table 5:** Height of anterior vertebral margin of patients in the two groups.

Group	Before the treatment	Difference before and after treatment		
		1 months	3 months	12 months
Group A	19.48 ± 4.35	1.38 ± 0.63^b^	1.36 ± 0.56^b^	1.15 ± 0.48^b^
Group B	19.52 ± 462	3.00 ± 1.22	3.72 ± 1.54	3.26 ± 1.64

*Note.* B refers to comparison with group B at the same time. (*P* < 0.05).

**Table 6:** Incidence of complications in the two groups (%).

Group	Recurrent vertebral fractures	Urinary tract infection	Pressure ulcers	Lung infection	The total infection rate
Group A	1	1	0	0	2 (4.00%)
Group B	1	2	3	2	8 (16.00%)

## Data Availability

The data used in the study are included within the article.
